This article has been retracted.

# Exploration of the Application Effect of the Darongtong Course Model Based on Deep Learning Enhancement in Nursing

**DOI:** 10.1155/2022/5484423

**Published:** 2022-08-25

**Authors:** Qi Han, Chunhua Ma, Ronghua Wang, Chen Xu

**Affiliations:** Shenzhen Polytechnic, Shenzhen 518055, China

## Abstract

In order to explore the application effect of the Darongtong course model based on deep learning enhancement in nursing, a total of 500 students in the school are investigated. The students in the contrast set are given the traditional teaching mode, and the students in the research set are provided with a teaching method based on deep learning-enhanced Darongtong mode. The evaluation results, teaching quality, students' cognition of teaching effect and their satisfaction with teaching mode before and after teaching were compared between the two groups. From the experimental results, it can be seen that the application of Datong general teaching based on deep learning in school nursing students can not only deepen students' understanding of theoretical knowledge, improve clinical skills, cultivate students' nurse patient communication skills and clinical thinking, but also improve students' subjective initiative. It is clearly evident that the Darongtong course model based on deep learning enhancement in nursing can stimulate students' interest in learning, and improve their self-study ability and problem-solving ability effectively.

## 1. Introduction

In 2017, the general office of the State Council pointed out in the opinions on deepening medical education cooperation and further promoting the reform and development of medical education that medical education and talent training should always be put in the first place in the development of health preservation. It is required to deepen the reform of medical education in Colleges and universities, and promote the combination of basic and clinical, clinical and prevention [1]. In addition, strengthen the general practice education for all medical students, standardize the management of clinical practice, and improve the ability of medical students to solve practical clinical problems [2]. Subsequently, in 2019, the State Council issued the “national vocational education reform implementation plan”, which proposed that higher vocational colleges should cultivate high-quality technical and skilled talents to serve regional development [3]. Under the medical model guided by professional needs, the health industry has developed rapidly and the supply of nursing talents is in short period. At the same time, the society continues to improve the requirements for the quality training of nursing talents, and the traditional training methods and curriculum models can no longer meet the needs of the times. Therefore, higher vocational colleges must explore innovative nursing talent training mode [4]. After 10 years of exploration, China has cultivated a number of high-quality nursing talents. Taking the nursing major of Shenzhen Vocational and Technical College as an example, the teaching reform practice of establishing the “Darongtong course model” has proved to be effective.

Deep learning refers to a learning method that can deeply understand and flexibly apply the knowledge learned and develop core literacy, with positive cognitive, metacognitive and non-cognitive inputs, and promote independent construction. Compared with deep-level processing learning, deep learning is an active learning method that seeks contact and understanding, models and evidence, including high-level cognition. In terms of learning results, deep learning can make students aware of their developmental understanding in the learning process, and actively participate in the course content with interest.

The rest of this paper is organized as follows: Section 2 demonstrates the related work. Then the research methods and observation indicators are presented in Section 3.  Section 4 presents the comparative results and analysis.  Section 5 concludes the paper.

## 2. Related work

The mode of inclusive curriculum is a comprehensive attempt of nursing teaching reform and a thorough reform of nursing curriculum mode in higher vocational colleges. It reflects the new requirements of the development of health industry for high-quality compound nursing talents in the new era [5]. The design of curriculum model is often based on constructivist learning theory, starting from needs and problems, to cultivate compound nursing talents with comprehensive nursing, traditional Chinese medicine nursing, elderly nursing, nutritional nursing and other qualities. Knowledge, technology, ability, quality and other aspects need to change from the previous single teaching mode to a comprehensive teaching mode. Through the integration of nursing environment, nursing evaluation, nursing diagnosis, nursing plan, nursing implementation and nursing evaluation, a curriculum structure throughout clinical work is established, so as to realize the great integration of learning fields. By reconstructing the learning situation, students can promote independent exploration and experience. This is conducive to the formation of a comprehensive integrated curriculum model of nursing majors jointly built by medical colleges. Constructivist learning theory emphasizes the interaction between external action field and students' internal knowledge experience. Learning is not only a process in which teachers impart knowledge to students, but also a process in which students actively construct their own knowledge and experience [6]. This theory is the basis of vocational education CBE courses, project courses, modular courses and learning field courses, which can broaden the theoretical vision of these courses and provide an important tool for the innovative implementation of comprehensive courses of nursing major in Higher Vocational Education [7].

The traditional teaching mode is mainly based on imparting and inculcating knowledge. Students are only regarded as passive knowledge recipients, emphasizing the memory, imitation and repeated practice of knowledge, which inhibits students' initiative and enthusiasm in learning [8]. This leads to a narrow range of students' knowledge, which is not conducive to students' extensive reading and thinking. In addition, theoretical knowledge is only a carrier without practical experience. Therefore, students cannot realize the “relevance” and “understanding” of cognition. It is difficult for medical students to care about diseases. Establish a holistic view and cultivate students' comprehensive working ability [9]. The content of basic courses is not embedded in the practical activities of completing nursing work, and cannot be effectively applied to practical work. Based on nursing environment, nursing evaluation, nursing diagnosis, nursing plan and nursing evaluation, the structure of comprehensive integrated curriculum is reconstructed. Starting with nursing problems, we should improve students' team teaching method through “explicit and implicit teaching method” and “vertical and horizontal teaching method”. Through standardized patients (SP) and other means, the introduction of clinical nursing ward round strategy, combined with psychological and emotional training, cultivate students' working ability [10]. It should be noted that there are differences in students' cognition of teaching quality and effect, especially in autonomous learning ability, nurse patient communication ability, teamwork ability, clinical thinking ability, problem solving ability and stimulating learning interest. The traditional curriculum structure is mainly based on “knowledge framework + knowledge symbols”, which can not connect the training links of nursing ability, and lack of activity design elements. It will result in the curriculum and clinical tasks are not relevant and incompatible. With the development of modern medicine, nursing work is more practical and professional, especially the high requirements of employers for “recruitment and use” [11]. This curriculum model leads to higher vocational students' theoretical and technical skills than undergraduates. The situation that students and both sides cannot reach the shore is not conducive to the cultivation of students' clinical ability [12]. On the other hand, based on constructivist learning theory, the in-depth learning and strengthening integration curriculum model aims to cultivate high-quality interdisciplinary nursing talents and establish a curriculum combining clinical work with nursing environment, nursing evaluation, nursing diagnosis, nursing plan and nursing evaluation. It forms a comprehensive curriculum model for nursing majors jointly built by medical schools, which directly connects students' school medical school learning path [13]. Since the social function of nursing is to promote the overall health of people's physiology, psychology and society, if higher vocational nursing ignores people's personality and integrity in teaching, then the curriculum is only related to objective knowledge, lacking emotion, procedure, method, and so on. If the characteristics of the social function (promoting health) of nursing specialty are ignored, students will not be able to enter the actual situation of nursing work. In addition, students do not know much about the characteristics of this major, and even have the view that “learning is useless” [14].

## 3. Research methods and observation indicators

### 3.1. General information

A total of 500 students are investigated in our school, and two nursing students who are about to enter clinical nursing courses from January 2021 to January 2022 are selected as participants, and a research group and a control group are carried out according to different classes. There are 40 students in each group. It is required that the classes of the subjects participating in the course are taught by the same instructor this semester, and the instructors of other courses use the same method to teach the two classes. They are randomly divided into a research group and a control group, with 40 students in each group. The students in the control group included 12 males and 28 females, aged 20-24 years old, with an average age of (21.45±3.26) years old, and the research group included 10 males and 30 females, aged 20-24 years old. The average age is (22.32±2.21) years old, and the general data such as age, gender and frequency of learning are compared between the two groups, *P*>0.05. There is no significant difference between the groups, and the comparison could be made, as shown in Figure 1 and Figure 2.

### 3.2. Research methods

#### 3.2.1. Curriculum Program

The students are given the traditional teaching mode, and the main contents are as follows: the teachers conducted relevant pre-job training for nursing students, and mainly carried out education and education to the trainees from the aspects of the hospital's department environment, characteristics, rules and regulations. And then the teacher will teach the students according to the syllabus of the internship and the teaching plan of the department, and do the assessment work before leaving the department.

To provide this set of students with a teaching method based on deep learning-enhanced Darongtong mode. The Darongtong course model breaks the usual “three-level” discipline barriers and is oriented to nursing positions. The core of medical basic courses and professional basic courses is to integrate content into professional courses, pay attention to the cultivation of humanistic care ability, and open new courses, including internal medicine patient care, surgical patient care, surgical patient care and other basic courses. Gynecological patient care, child care, clinical nursing integration and nursing application technology, each new course has a project proposal for the course structure. Each program analyzes typical work tasks and the ability to perform work tasks according to the nursing profession, and then derives appropriate learning tasks from the work tasks, develops learning goals, and determines teaching. Plan and design classrooms, plan a variety of course evaluation methods, and implement the connection between nursing courses and work tasks.

In addition, the “Great Rongtong” curriculum model changes the goal of talent training from the traditional focus on knowledge base to focus on knowledge application, that is, comprehensive skills training. By analyzing the basic concepts and principles of the curriculum and classifying its relevance to nursing tasks, the curriculum structure is reconstructed from the original “knowledge frame+knowledge symbols” to “task frame+symbols+steps”. The multi-dimensional and three-dimensional correlation of theoretical knowledge related to pathological changes, disease process, treatment and nursing corresponds to human body functions and pathological changes of patients, from pathological changes of patients to clinical manifestations and treatment principles to pathological changes. The principle of treatment should take appropriate nursing measures, change the subject curriculum into an active curriculum, and earnestly implement the commitment of nursing tasks. Further, objective knowledge and subjective knowledge are combined into specific steps to realize the effective connection between learning and nursing work. In addition, under this mode of teaching, the holistic view of human physiology, psychology and society is emphasized, and social emotions, procedures and methods are linked with “ladder symbols” to carry out holistic nursing training. At the same time, aiming at the lack of social emotion and specific operation steps in psychological nursing in subject textbooks, to solve the problem that psychological nursing descriptions in traditional textbooks only have one sentence or knowledge symbols that are difficult to implement, teach students to observe and analyze typical work situations by simulating, in order to solve the problem of patients. Finally, it is necessary to analyze and discuss typical cases before class to give students a preliminary understanding of the disease. The teacher summarizes and analyzes the problems existing in the pre-class discussion, and explains the etiology, pathogenesis, clinical characteristics, diagnosis and treatment of the disease. It can realize the communication between teachers and students and between students and students, exercise students' clinical thinking ability, and enable students to firmly grasp the knowledge points they have learned. In clinical teaching, the students should pay more attention to ask standardized patients or patients' medical history, and carry out physical examination and relevant skill operations, and carry out relevant auxiliary examinations, so that students can make their own diagnosis and formulate treatment plans.

#### 3.2.2. Data collection methods

This research is conducted with the help of the Questionnaire Star App [15]. The subjects' class sets are explained before and after the course study. The main contents are the purpose of the survey and filling-in requirements. Students scanned the QR code in the set to fill in by themselves. The survey data is exported from the Star App, and the members of the research team screen the questionnaires according to the students' fill-in.

### 3.3. Observation indicators

#### 3.3.1. Contrast of the two sets of students' scores before and after teaching

The assessment results include theoretical basis, clinical operation ability, Case analysis and nursing analysis Each item is scored from 1 to 50 points, with a total of 100 points. The higher the score is, the better the teaching effect will be. The assessment results are jointly assessed by 2 teachers in the same department who did not participate in the study.

#### 3.3.2. Comparing the evaluation of the two sets of students on the quality of this teaching

Refer to the standards in the DREEM scale to investigate the teaching quality [16]. The table consists of following parts: learning perception, perception of teachers, teaching self-perception, environmental perception and social self-perception. The higher the total score is, the better the teaching quality will be.

#### 3.3.3. Comparing the two sets of students' recognition of the teaching effect

Questionnaire issued by the Science and Education Division, including the following questions: Through this teaching, have you improved your self-learning ability, nurse-patient communication ability, teamwork ability, clinical thinking ability, problem-solving ability and arousing interest in learning, each question option Divided into yes or no, the higher the proportion of choosing “yes”, the higher the students 'recognition of the teaching effect.

#### 3.3.4. Contrast of the two sets of students' evaluation of the results of the objective structural clinical ability test

Comparing the evaluation of the two groups of students on the objective structural clinical ability test, The specific contents include: collecting medical history; physical examination; using diagnostic auxiliary examination; diagnostic ability; making medical decision-making ability; implementing medical decision-making ability; continuing medical decision-making ability; continuing Treatment and nursing ability; correctly handle the doctor-patient relationship.

The emphases of this study include: helping students master theoretical knowledge comprehensively, broadening the scope of knowledge, helping the application of knowledge, and closely combining basic knowledge with clinical skills; Improve self-learning ability, exercise the ability to independently consult literature, acquire information, improve the ability to analyze and solve problems, and improve the ability of comprehensive analysis, logical thinking and teamwork; Improve the expression ability and learn to communicate effectively with others. The research objects include students, teachers, patients and other cases.

#### 3.3.5. Comparing the two sets of students' satisfaction with the teaching mode

The nursing satisfaction survey scale developed by the hospital is used to investigate the teaching quality, teaching environment and teaching content. The scale includes a total of 4 options, namely very satisfied, satisfied, average and dissatisfied. The calculation of total satisfaction can be defined as: (Number of very satisfied cases + Number of satisfied cases + Number of general cases)/ Total number of students × 100%.

### 3.4. Statistical methods

All the data are organized, and a corresponding database is established for it, and all the databases are entered into SPSS 26.0 for data processing, and the measurement data is tested for normality, expressed as (x±s), and between-set data Independent samples t test is used, paired samples t test is used for intra-set data, and Mann-Whitney U test is used for non-normality; the rate is expressed as%, and the test is *χ*^2^; when P < 0.05, the difference between the data is considered to be statistically large.

## 4. Comparative results and analysis

### 4.1. The assessment scores and total scores of the two sets of students before and after teaching

Before teaching, the scores of students in the two sets in theoretical basis, clinical operation ability, case analysis and nursing analysis are all lower, and there is no large difference (*P* > 0.05). The scores of students in the research set are notoriously higher than those in the contrast set (*P* < 0.05), as shown in Table 1. In Table 1, the symbol ^∗^ indicates that contrast with before teaching, P < 0.05, the difference is statistically large.

### 4.2. Contrast of DREEM scale data of two sets of students

After the teaching, there are differences in the evaluation of the teaching quality of the two sets of students, among which the scores of students' perception of learning and self-cognition of teaching in the research set are notoriously higher than those in the contrast set (*P* < 0.05), and there is no large difference in other teaching quality evaluations (*P* > 0.05), as shown in Table 2.

### 4.3. Contrast of two sets of students' evaluation of teaching effect

After the teaching, there are differences in the recognition of the teaching quality effect by the students in the two sets. The students in the research set had notoriously higher recognition of autonomous learning ability, nurse-patient communication ability, teamwork ability, clinical thinking ability, problem-solving ability and stimulating learning interest.  Table 3 shows the degree of recognition of the two sets of regular trainees for the quality of the teaching effect.

### 4.4. Contrast of the evaluation results of the objective structural clinical ability test between the two sets of students

After the teaching, there are large differences in the evaluation of the results of the objective structural clinical ability test by the two sets of students. The evaluation effects of improving comprehensive analysis, logical thinking ability, teamwork spirit, improving expression ability, learning to communicate effectively with others, and communication are all notoriously better than those of the contrast set (*P* < 0.05), as shown in Table 4.

### 4.5. Contrast of two sets of students' satisfaction with the teaching mode

There are large differences in the satisfaction of the two sets of students with the teaching mode in this study, and the total satisfaction of the research set is notoriously higher than that of the contrast set (*P* < 0.05), as shown in Table 5.

## 5. Conclusions

In this study, the exploration of the application effect of the Darongtong course model based on deep learning enhancement in nursing is conducted. From the results, it can observed that the application of deep learning-based Darongtong teaching to nursing students in school can deepen students' understanding of theoretical knowledge, improve clinical skills and cultivate students' nurse-patient communication skills and clinical thinking. Also, it is beneficial of improving students' understanding of theoretical knowledge. It shows that giving full play to students' subjective initiative and stimulating learning interest can improve their autonomous learning ability and problem-solving ability. The above model plays a good role in cultivating students' lifelong learning spirit and promoting medical progress [5].

## Figures and Tables

**Figure 1:** Analysis of the total sample size of school students.

**Figure 2:** Frequency of Acceptance Learning.

**Table 1:** Contrast of the assessment scores and total scores of the two sets of students before and after teaching.

Entry		Contrast set (*n* = 40)	Study set (*n* = 40)	*T*	*P*
Theoretical basis	Before teaching (points)	11.23 ± 3.62	12.37 ± 2.86	−0.605	0.558
	After teaching (points)	16.50 ± 3.26^∗^	22.57 ± 3.36^∗^	−3.307	0.008

Clinical skills	Before teaching (points)	12.56 ± 3.56	11.95 ± 2.21	0.357	0.729
	After teaching (points)	15.86 ± 4.26^∗^	23.32 ± 3.65^∗^	−3.507	0.009

Case analysis	Before teaching (points)	11.50 ± 3.02	11.69 ± 3.45	−0.35	0.819
	After teaching (points)	17.96 ± 3.17^∗^	22.89 ± 2.01^∗^	−3.217	0.009

Nursing analysis	Before teaching (points)	10.57 ± 3.12	11.65 ± 3.39	−0.574	0.579
	After teaching (points)	18.93 ± 4.29^∗^	24.10 ± 2.16^∗^	−2.637	0.05

Overall result	Before teaching (points)	45.50 ± 3.69	44.02 ± 3.87	0.563	0.586
	After teaching (points)	79.26 ± 5.39^∗^	92.66 ± 6.52^∗^	−3.88	0.003

**Table 2:** The evaluation effect of the two sets of students on the quality of this teaching.

Set	Learning perception (points)	Perception of the teacher (points)	Teaching self-perception (points)	Awareness of the environment (points)	Social self-perception (points)
Contrast set (*n* = 40)	30.26 ± 3.57	32.57 ± 4.21	24.57 ± 3.59	33.56 ± 4.36	32.59 ± 4.68

Study set (*n* = 40)	45.50 ± 5.89	33.26 ± 5.50	40.26 ± 5.67	34.05 ± 4.53	33.57 ± 4.26

*T*	−5.331	−0.501	−5.727	−0.191	−0.379

*P*	＜0.001	0.807	＜0.001	0.852	0.712

**Table 3:** The degree of recognition of the two sets of regular trainees for the quality of the teaching effect.

Set	Self-learningability		Nurse-patientcommunication skills		Team work		Clinicalthinking skills		Problem solving skills		Stimulate interest in learning	
	Yes	No	Yes	No	Yes	No	Yes	No	Yes	No	Yes	No
Contrast set (*n* = 40)	13	27	15	25	13	27	17	23	21	19	17	23
Study set (*n* = 40)	35	5	37	3	30	10	37	3	35	5	33	7
*Χ^2^*	25.208		26.593		14.532		22.792		11.667		13.653	
*P*	＜0.001		＜0.001		＜0.001		＜0.001		0.001		0.001	

**Table 4:** Contrast of the evaluation results of the objective structural clinical ability test by the two sets of students.

Content	Contrast set (*n* = 40)	Study set (*n* = 40)	*Χ^2^*	*P*
Contribute to a comprehensive grasp of theoretical knowledge	15	37	26.593	＜0.001
Broaden their knowledge	13	30	14.532	＜0.001
Contribute to knowledge application, making basic knowledge and clinical skills closely integrated	12	37	32.916	＜0.001
Improve independent learning ability	11	36	32.237	＜0.001
Exercise the ability to independently access literature and materials and hand over information	12	37	32.916	＜0.001
Improve analytical and problem-solving skills	11	38	38.394	＜0.001
Improve the ability of comprehensive analysis and logical thinking	12	37	32.916	＜0.001
Spirit of cooperation	13	34	22.747	＜0.001
Improve expressiveness	11	32	22.175	＜0.001
Learn to communicate effectively with others, including classmates, teachers, and patients	14	35	23.226	＜0.001

**Table 5:** Contrast of the satisfaction of the two sets of students with the teaching mode (*n*/%).

Set	Very satisfied	Satisfy	Generally	Dissatisfied	Total satisfaction
Contrast set (*n* = 40)	10	7	4	21	19 (47.50)
Study set (*n* = 40)	20	15	3	2	35 (87.50)
*Χ* ^2^					14.587
*P*					＜0.001

## Data Availability

The simulation experiment data used to support the findings of this study are available from the corresponding author upon request.
